# Study on the Mechanism of Qigu Capsule in Upregulating NF-*κ*B/HIF-1*α* Pathway to Improve the Quality of Bone Callus in Mice at Different Stages of Osteoporotic Fracture Healing

**DOI:** 10.1155/2021/9943692

**Published:** 2021-09-13

**Authors:** Peige Wang, Jie Ding, Guangyue Yang, Wen Sun, Hailing Guo, Yongfang Zhao

**Affiliations:** ^1^Shi's Center of Orthopedics and Traumatology, Shuguang Hospital Affiliated to Shanghai University of Traditional Chinese Medicine, Shanghai 201203, China; ^2^Institute of Traumatology & Orthopedics, Shanghai Academy of Traditional Chinese Medicine, Shanghai 201203, China

## Abstract

**Objective:**

The present study intends to investigate the effects and underlying molecular mechanism of Qigu Capsule (QG) on fracture healing in mice with osteoporosis.

**Methods:**

Ten-week-old female C57BL/6 mice were ovariectomized and three weeks later were evaluated for successful modeling. Then, all mice were prepared into models of transverse fracture in the right middle femoral shaft. Mice were treated daily using a gavage with normal saline (the NS group), Qigu Capsule (the QG group), or alendronate (the ALN group) postoperatively. Fracture callus tissues were collected and analyzed by X-ray, micro-CT, western blot (WB), and transmission electron microscope (TEM) on postoperation Day 14 (POD14), POD28, and POD42.

**Results:**

(1) X-ray results showed that on POD14, the QG group had the fracture healing score significantly higher than the NS and ALN groups, and on POD28, it had the fracture healing score higher than the NS group, suggesting that QG could promote fracture healing. (2) Micro-CT results showed that on POD14, the QG group had tissue bone density (TMD) significantly higher than the NS and ALN groups, and on POD28 and POD42, it had bone volume fraction, trabecular number, and TMD significantly higher than the NS group. (3) WB results showed that, compared with the NS group, the QG group had significantly increased expression of nuclear factor kappa-B (NF-*κ*B), hypoxia-inducible factor-1*α* (HIF-1*α*), bone alkaline phosphatase (BALP), runt-related transcription factor 2 (Runx2), bone Gla protein (BGP) and collagen I*α*1 (COLI*α*1) on POD14, significantly increased expression of NF-*κ*B, HIF-1*α*, BALP and COLI*α*1 on POD28, and significantly increased expression of NF-*κ*B, HIF-1*α*, and Runx2 on POD42. (4) TEM scanning results showed that, compared with the NS and ALN groups, the QG group had significantly increased numbers of autophagic vacuoles (AVs) in osteocytes on POD14, POD28, and POD42.

**Conclusion:**

QG could accelerate osteoporotic fracture healing by promoting bone formation and osteocyte autophagy, possibly through upregulating the NF-*κ*B/HIF-1*α* signaling pathway.

## 1. Introduction

With the population aging, fragility fracture has become a worldwide disease [1]. It is the most serious consequence of osteoporosis, a systemic skeletal disease characterized by low bone mass and microarchitectural deterioration of bone tissue that cause an increase in bone fragility [2]. Fragility fracture may occur in almost all skeletal segments, and it mostly occurs in the vertebrae, proximal femur and humerus, and distal radius [1]. Studies have shown that osteoporosis may delay fracture healing and reduce the biochemical properties of bone, and the risk of bone nonunion and death after fragility fracture is increasing [3–5]. Therefore, the prevention and treatment of fragility fracture tend to be a hot research topic and bottleneck in current studies.

It has been proposed in relevant guidelines that the prevention and treatment of fragility fracture should focus on intervention of the primary disease, enhancement of bone mineral density (BMD), and prevention of refracture [1]. Anti-bone-resorptive drugs, such as alendronate, are usually used to prevent and treat fragility fracture because they can promote fracture healing by inhibiting the activity of osteoclasts [6, 7]. However, studies also show that bisphosphonate may increase the risk of delayed fracture healing [8]. According to a study, traditional Chinese medicine (TCM) compounds for kidney reinforcing have confirmed efficacy in preventing and treating fragility fracture, and they can increase BMD and improve bone metabolism and bone turnovermarkers in patients with osteoporosis [9]. In addition, animal experiments demonstrate that TCM compounds for kidney reinforcing act against osteoporosis significantly, the mechanism of which involves multiple regulatory pathways [10].

Qigu Capsule (QG), composed of Herba Epimedium, prepared *Polygonum multiflorum*, *Astragalus membranaceus*, *Dendrobium*, Herba Cistanches, Rhizoma Drynariae, and *Chrysanthemum*, is a TCM compound for kidney reinforcing to treat postmenopausal osteoporosis and has been granted the National New Drug License (National Drug License No. Z20090039). A series of studies have been carried out on its clinical application and basic research. According to the preliminary study of the research group, QG could significantly increase BMD in patients with osteoporosis with the BMD of lumbar vertebrae and femoral neck in patients increasing by 2.7% and 4.5%, respectively, after 24 months of QG treatment compared with the control group [11]. Also, QG could promote fracture healing and improve the clinical symptoms of postmenopausal osteoporotic fracture induced by vertebral compression [12]. In in vivo studies, QG could enhance bone strength in rats with osteoporosis and promote fracture healing in mice with postmenopausal osteoporosis by improving bone microstructure and biomechanical properties [13, 14]. In in vitro studies, QG could not only promote osteoblasts proliferation, improve the alkaline phosphatase activity of osteoblasts, and increase the number of mineralized nodules but also inhibit the number, the area, and the depth of bone resorption lacuna of osteoclasts to certain degrees. Furthermore, QG could significantly downregulate the expression of receptor activator of NF-*κ*B ligand (RANKL), upregulate the expression of osteoprotegerin (OPG) mRNA, and slightly downregulate the expression of receptor activator of NF-*κ*B (RANK) mRNA [15–17]. However, the underlying molecular mechanism of QG on osteoporotic fracture healing is required to be further studied.

Hypoxia-inducible factor-1*α* (HIF-1*α*) is a core transcription factor that regulates intracellular environment and homeostasis under hypoxia. Hypoxia can activate HIF-1*α* expression [18]. Rupture of blood vessels and hematoma formation at the fracture site can lead to local hypoxia, so HIF-1*α* may play an important role in fracture healing according to a study [19]. Under hypoxia conditions, HIF-1*α* can promote the expressions of runt-related transcription factor 2 (Runx2), bone alkaline phosphatase (BALP), and bone Gla protein (BGP) and regulate bone formation by enhancing the bone formation function of osteoblasts [20]. At the fracture end, HIF-1*α* regulates osteocyte autophagy to promote fracture healing [21, 22]. Nuclear factor kappa-B (NF-*κ*B), which is often activated in inflammatory diseases, is an inflammatory transcription factor [23, 24]. In the skeletal system, inflammation is closely related to a number of bone diseases, including fracture, nonunion, and osteoporosis, while acute inflammation is a key step in bone healing and bone remodeling. NF-*κ*B can regulate the inflammatory response in bone formation, bone resorption, and bone remodeling [25]. A study has shown that HIF-1*α* and NF-*κ*B interfere with each other, and NF-*κ*B regulates HIF-1*α*. In the event of NF-*κ*B deficiency, HIF-1*α* cannot be effectively transcribed [26]. Therefore, the NF-*κ*B/HIF-1*α* pathway may play an important role in the process of fracture healing.

Thus, we hypothesized that QG would accelerate osteoporotic fracture healing by promoting bone formation via activation of the NF-*κ*B/HIF-1*α* signaling pathway. To test this, mouse osteoporotic fracture models were developed in the present study to investigate the role of QG in repairing osteoporotic fracture and quality of bone callus, local expressions of key proteins, and osteocyte autophagy at the fracture site were examined in vivo.

## 2. Materials and Methods

### 2.1. Experimental Animals

A total of 72 ten-week-old C57/BL6 female mice were provided by the Laboratory Animal Center of Shanghai University of Traditional Chinese Medicine (Laboratory Animal License No. SYK (Shanghai) 2014-0008). All mice were maintained in a well-ventilated room at 25°C on a 12°h light/dark cycle and allowed free access to water and food. The animal experiment was approved by the Institutional Animal Care and Use Committee of Shanghai University of Traditional Chinese Medicine in accordance with the National Institute of Health Guidelines.

### 2.2. Development of Mouse Osteoporotic Fracture Models

The mice were anesthetized by intraperitoneal injection of 1% pentobarbital sodium (10 mg/kg) and received bilateral oophorectomy through a dorsal incision. Three weeks after the operation, all mice were prepared into models of transverse fracture in the right middle femoral shaft following the scheme proposed by Diwan et al. [27]. Anesthesia was induced with 1% pentobarbital sodium (10 mg/kg) via intraperitoneal injection. After shaving the fur and disinfecting the skin, a 1 cm incision was cut on the lateral right femur to expose the middle femur. A circular saw of 0.15 mm in thickness was used on a dental microelectric motor (Strong 102, SAESHIN, KR) to cause a fracture in the middle femur in the mouse, and then a stainless steel nail of 0.45 mm in diameter was inserted into the bone marrow cavity of the femur for fixation. The animals were monitored for general postsurgical health and function of the fractured limb.

### 2.3. Experimental Grouping and Administration

The modeled mice were grouped into the NS group (24 mice), the QG group (24 mice), and the ALN group (24 mice) by the random number table method. They were administrated the dose of an equivalent effect in humans by body surface area. The NS group was given saline (0.5 ml/mouse, once per day), the QG group was given QG (Xiamen Chinese Medicine Factory, 0.636 mg/g body weight, 0.5 ml/mouse, once per day), and the ALN group was given alendronate sodium (Hangzhou MSD, 0.00895 mg/g body weight, 0.5 ml/mouse, once per week). One day after fracture modeling, gavage treatment was started in the mice. On postoperation Day 14 (POD14), POD28, and POD42, 8 mice were taken from each group at each time point and were sacrificed by cervical dislocation following anesthesia by intraperitoneal injection of 1% pentobarbital sodium (10 mg/kg). Then, all mice were placed inside a small animal X-ray machine to observe the degree of fracture healing at the fracture end in the femur. After that, the right femur was taken out, and the muscle tissue was removed. Samples for micro-CT scanning were stored in 75% alcohol, those for transmission electron microscope (TEM) scanning were fixed in 2.5% glutaraldehyde, and those for western blot (WB) detection were stored at −80°C.

### 2.4. X-Ray Scanning

A small animal X-ray machine (Faxitron X-Ray Corp, Wheeling, IL) was used to perform X-ray scanning on the right fractured femur at exposure time of 1.5 seconds and voltage of 28 kV. Following the scheme proposed by Shuid et al., the radiological scoring criteria were used to evaluate the staging of fracture healing [28]. Two experienced researchers scored the degree of fracture healing according to X-ray findings using the blind method.

### 2.5. Micro-CT Scanning

The micro-CT system (SkyScan 1276, Bruker, USA) was used to scan the fractured femur on POD14, POD28, and POD42, with the long axis of the femur aligned with that of the scanner. Parameters of the scanning system were set as 80 kV, 80 *μ*A, and 2,960 ms exposure time, and the isotropic voxel size was set as 12 *μ*m. After scanning, the site of the new bone callus was displayed in the micro-CT software, and tissue mineral density (TMD), total bone volume (TV), bone volume fraction (BV/TV), and mean trabecular number (Tb. N) of the bone callus were analyzed.

### 2.6. Western Blot Detection

The femoral callus tissue of each mouse was ground into powder in liquid nitrogen, and then the RIPA lysis buffer containing protease inhibitor was added. After the mixture was centrifuged at 4°C and 12,000 rpm for 20 minutes, the supernatant was collected. The protein sample was separated by SDS-PAGE and then transferred to a polyvinylidene fluoride (PVDF) film. The membrane was incubated in TBST buffer with 5% bovine serum albumin at room temperature for 1 hour and followed by incubation with anti-NF-*κ*B (1 : 500, rabbit, ab209795, Abcam), anti-HIF-1*α* (1 : 1000, mouse, ab113642, Abcam), anti-BALP (1 : 500, rabbit, ab108337, Abcam), anti-BGP (1 : 200, rabbit, ab93876, Abcam), anti-Runx2 (1 : 1000, mouse, ab76956, Abcam), anti-collagen I*α*1 (COLI*α*1) (1 : 1000, mouse, ab88147, Abcam), anti-COLI*α*2 (1 : 500, rabbit, ab96723, Abcam), and anti-*β*-actin (1 : 1000, mouse, ab8226, Abcam) overnight at 4°C. Next, the membrane was incubated with secondary antibodies (1 : 1000, Byotime) at room temperature for 1 hour. The signal was detected by an enhanced chemiluminescence kit (BeyoECL Star, P0018A, Byotime). Quantitative analysis was performed using the ImageJ software.

### 2.7. Transmission Electron Microscope Scanning

Each TEM sample was taken from the femoral callus, fixed in 2.5% glutaraldehyde for 24 hours, decalcified in 5% EDTA for 4 weeks, cut into 1 mm^3^ pieces. Then, the sample was rinsed with 0.1 mol/L PBS (pH = 7.2) 4 times and for 45 minutes/time, fixed in 1% elemental acid (0.2 mol/L PBS at 1 : 1 ratio) for 4 hours, and rinsed with PBS 3 times and for 15 minutes/time. Then, the sample was dehydrated with 30%, 50%, 70%, and 90% ethanol, a mixture of 90% ethanol and 90% acetone at 1 : 1 ratio, 90% acetone, and 100% acetone and in turn fully soaked in 618 epoxy embedding liquid. After that, the sample was transferred to a special embedding plate, embedded at 37°C overnight, and then polymerized in the embedding reagent at 60°C for 48 hours. The Leica 705902 ultra-thin slicer was used to cut the sample into slices of 70 nm in thickness. In the end, the sample was stained with uranium dioxide acetate and lead citrate and observed under a Philip Tecnai-12 TEM at the accelerating voltage of 80 kV.

### 2.8. Statistical Analysis

All data were presented as mean ± SD. Data were analyzed by one-way analysis of variance (ANOVA) with LSD-t's multiple comparisons, using statistical software SPSS 19.0 (SPSS Ltd., Chicago, IL, USA). *P* < 0.05 or *P* < 0.01 is considered statistically significant.

## 3. Results

### 3.1. Effect of QG on Osteoporotic Fracture Healing

X-ray scoring of the fracture showed that on POD14, both the QG group and the ALN group had the fracture healing score higher than the NS group, with the difference of statistical significance (*P* < 0.05) and the QG group had the fracture healing score higher than the ALN group (*P* < 0.05); on POD28, both the QG group and the ALN group had the fracture healing score higher than the NS group, with the difference of statistical significance (*P* < 0.05); and on POD42, there was no significant difference in fracture healing score between the three groups (Figure 1(b)). Such results suggested that QG could promote osteoporotic fracture healing.

### 3.2. Effect of QG on Local Bone Microstructure in Osteoporotic Fracture

Micro-CT results showed that on POD14, the QG group had TMD significantly higher than the NS group and the ALN group (*P* < 0.05) while there were no statistically significant differences in TV, BV/TV, and Tb. N between the three groups (*P* > 0.05); on POD28 and POD42, the QG group and the ALN group had significant high BV/TV (*P* < 0.01) and also had significantly high TMD and Tb. N (*P* < 0.05) compared with the NS group (Figures 2(b)–2(e)). Such results suggested that QG could improve local TMD and improve bone microstructure in osteoporotic fracture.

### 3.3. Effect of QG on NF-*κ*B and HIF-1 Expressions

Results showed that on POD14, POD28, and POD42, QG could significantly promote NF-*κ*B and HIF-1 expressions compared with the NS group (*P* < 0.05, Figures 3(b) and 3(c)), while in the ALN group, NF-*κ*B and HIF-1 expressions were not affected (Figures 3(b) and 3(c)). Such results suggested that QG could promote fracture healing by enhancing NF-*κ*B and HIF-1 expressions.

### 3.4. Effect of QG on BALP, BGP, and Runx2 Expressions

Results showed that compared with the NS group, the QG group had significantly increased BALP, BGP, and Runx2 expressions on POD14 (*P* < 0.05, Figures 4(b)–4(d)), significantly increased BALP expression on POD28 (*P* < 0.05, Figure 4(b)), and significantly increased Runx2 expression on POD42 (*P* < 0.05, Figure 4(d)), while there were no statistically significant differences in BALP, BGP, and Runx2 expressions between the ALN group and the NS group at these three time points (*P* > 0.05, Figures 4(b)–4(d)). Such results suggested that QG could promote bone formation by enhancing the expression of marker proteins of bone formation in callus.

### 3.5. Effect of QG on COLI*α*1 and COLI*α*2 Expressions in Extracellular Matrix

Results showed that compared with the NS group, the QG group had significantly upregulated CoLI*α*1 expression on POD14 and POD28 (*P* < 0.05, Figure 5(b)) while there were no statistically significant differences in CoLI*α*1 and CoLI*α*2 expressions between the ALN group and NS group at the three time points (Figures 5(b) and 5(c)). Such results suggested that in the process of fracture healing, QG could promote the expression of extracellular matrix proteins.

### 3.6. Effect of QG on the Number of Autophagic Vacuoles

TEM scanning results showed typical autophagic vacuoles (AVs) in bone callus in mice with osteoporotic fracture in different groups and that the QG group had more AVs than the NS and ALN groups on POD14, POD28, and POD42 (Figures 6(a) and 6(b)). According to the AV count analysis, the QG group had significantly more AVs than the NS and ALN groups on POD14, POD28, and POD42 (*P* < 0.05, Figure 6(c)), while there was no statistically significant difference between the ALN group and the NS group (*P* > 0.05, Figure 6(c)). Such results suggested that QG could increase the number of AVs in osteocytes in the process of osteoporotic fracture healing and might promote osteocyte autophagy.

## 4. Discussion

The objective of this study was to analyze the effects of clinical dosage of QG, given at different time points, on osteoporotic fracture healing. According to the X-ray scoring and micro-CT findings, on POD14, the QG group had the fracture healing score and TMD significantly higher than the NS group and the ALN group. Moreover, on POD28 and POD42, the callus microstructure in the QG group further improved, as indicated by the fact that BV/TV, TMD, and Tb. N were all significantly increased compared to the NS group. The early stage of fracture repair encompasses primary bone formation (synthesis by mature osteoblasts or osteoprogenitors), chondrocyte proliferation, hypertrophy, and mineralization [29]. In addition, calcification of fibrocartilage calluses was completed within 3-4 weeks of normal fracture in rodents and was followed by initial bony union [30]. Based on the above, we concluded that QG improved the quality of bone callus at different stages of osteoporotic fracture healing. Especially QG enhanced callus growth and mineralization and the subsequent transformation of fibrocartilage callus into woven bone during the early stage of osteoporotic fracture healing.

Blood shortage and reduced oxygen supply induced by fracture cause the activation of HIF-1*α*, an oxygen-sensitive transcription factor that mediates cellular responses to hypoxia during the pathological process of many diseases [31]. Komatsu and Hadjiargyrou built rat femoral fracture models and collected bone callus samples on POD3, POD5, POD7, POD10, POD14, and POD21 after fracture. At all the time points, they observed upregulated HIF-1*α* expression in bone callus, which peaked on POD10 [32]. In the present study, postfracture HIF-1*α* expression level in bone callus was detected. Compared with the NS group, the QG group had HIF-1*α* expression significantly upregulated on POD14, POD28, and POD42, suggesting that QG could promote HIF-1*α* expression in bone callus. Between the NS group and the ALN group, there were no significant differences in HIF-1*α* expression on POD14, POD28, and POD42, but HIF-1*α* expression decreased with the progression of fracture healing, suggesting that HIF-1*α* expression might first increase and then decrease during fracture healing. According to X-ray and micro-CT findings, QG could accelerate fracture healing by enhancing bone formation earlier and improving TMD, suggesting that QG might speed up osteoporotic fracture healing by promoting HIF-1*α* expression.

In the event of a fracture, osteoblasts play an irreplaceable role in fracture healing [33]. Previous studies show that HIF-1*α* can regulate the function of osteoblasts. According to Xu et al., HIF-1*α* could promote Runx2 expression and regulate early bone formation under hypoxia conditions [34]. According to Huang et al., the use of hypoxia simulator COCL2 to treat tibial fracture in rats could promote the expressions of HIF-1*α* and its downstream factors Runx2, ALP, and BGP to enhance tibial fracture healing [21]. In the present study, osteogenic genes were detected, the results of which showed that compared with the NS group, the QG group had significantly increased expression of BALP, BGP, Runx2, and COLI*α*1 on POD14, significantly increased expression of BALP and COLI*α*1 on POD28, and significantly increased expression of Runx2 on POD42. Such findings suggested that QG might promote bone formation by upregulating HIF-1*α* expression to accelerate fracture healing.

According to recent studies, the signal transduction of NF-*κ*B and HIF-1*α* influences and depends on each other. NF-*κ*B is a transcriptional activator of HIF-1*α*, and the baseline activity level of NF-*κ*B is a prerequisite for HIF-1*α* accumulation under normoxia and hypoxia conditions [35]. Besides, HIF-1*α* and NF-*κ*B were activated almost at the same time. For example, IL-1*β* upregulates HIF-1*α* expression under normoxia conditions and activates the expression of HIF-1*α*-dependent VEGF, which requires the involvement of NF-*κ*B [35]. NF-*κ*B expression was also detected in the present study. Compared with the NS group, on POD14, POD28, and POD42, the QG group had significantly upregulated expression of NF-*κ*B, which might be related to the activation of HIF-1*α* and suggested that QG might promote fracture healing by enhancing bone formation through the NF-*κ*B/HIF-1*α* signaling pathway.

Autophagy is an evolutionarily conserved intracellular process, in which domestic cellular components are selectively digested for the recycling of nutrients and energy. This process is indispensable for cell homeostasis maintenance and stress responses [36]. It has been found in studies in recent years that osteocyte autophagy plays an important role in bone homeostasis and can promote fracture healing. Moreover, autophagy is believed to be a HIF-1*α*-dependent adaptive metabolic response to hypoxia [37–39]. Qiao et al. reported that HIF-1*α* might play an essential role in fracture healing by upregulating osteocyte autophagy [22]. The effect of OG on local osteocyte autophagy in fracture was observed in the present study. Osteocyte autophagy in bone callus detected by TEM scanning showed that QG increased the number of AVs in osteocytes during fracture healing on POD14, POD28, and POD42. According to a previous study, HIF-1*α* could promote fracture healing by upregulating osteocyte autophagy, and inhibition of HIF-1*α* could cause osteocyte autophagy to decline and thus inhibit fracture healing in rats [21]. Besides, osteocyte autophagy is closely related to the differentiation and mineralization of osteoblasts, and the conditioned loss of osteocyte-specific ATG7 affects osteocyte autophagy and thereby inhibits bone formation and leads to bone loss [40]. Apatite crystals detected in autophagy vacuoles indicate a close association between autophagy and bone mineralization, and inhibition of autophagy stops outward mineral transport from osteoblasts [41]. In the present study, the significantly increased number of AVs in osteocytes in the QG group suggested that QG might promote fracture healing by enhancing bone formation through upregulating osteocyte autophagy, which should be further studied in the future.

There are some limitations to this work. First, the influence of the systematic administration of QG on other tissues and organs should be thoroughly assessed to determine its potential adverse effects. Fortunately, no abnormal behaviors or health conditions were observed in any of the animals in the present study. Second, in the present study, we analyzed only one dosage of QG. It is possible that modifying the dosage or treatment duration may enhance osteoporotic fracture healing, although the positive effects of QG were substantial at this dosage. In addition, fracture healing is an integrated process that involves multiple types of cells and is a carefully organized process between the formation of new bone tissue by osteoblasts and the resorption of cartilage and bone by osteoclasts; therefore, it would be interesting to further explore the roles of osteoblasts and osteoclasts in bone callus formation and remodeling during QG treatment. Finally, extensive clinical application of QG makes it possible to do some clinical studies on QG. In this situation, we may have a more profound understanding of the role of QG in osteoporotic fracture healing.

## 5. Conclusion

Taken together, the present results indicated that QG could improve the quality of bone callus at different stages of osteoporotic fracture healing and particularly promote fracture healing at the early stage by enhancing bone formation and osteocyte autophagy via the NF-*κ*B/HIF-1*α* pathway. However, such results require further research, and the mechanism involved requires to be explored in order to further enrich the theoretical connotation of the treatment of osteoporotic fracture with TCM compounds for kidney reinforcing.

## Figures and Tables

**Figure 1:** Effect of QG on X-ray scoring in mice with osteoporotic fracture. (a) X-ray images of the fracture in the middle femur of the three groups on POD14, POD28, and POD42; (b) fracture healing scores of the three groups on POD14, POD28, and POD42. Compared with the NS group, ^*∗*^*P* < 0.05; compared with the ALN group, ^*#*^*P* < 0.05.

**Figure 2:** Effect of QG on local bone microstructure in mice with osteoporotic fracture. (a) 3D images of local bone callus in fracture; (b) TV; (c) BV/TV; (d) TMD; (e) Tb. N. Compared with the NS group, ^*∗*^*P* < 0.05, ^*∗∗*^*P* < 0.01; compared with the ALN group, ^*#*^*P* < 0.05.

**Figure 3:** Effect of QG on NF-*κ*B and HIF-1 expressions in bone callus tissue in mice with osteoporotic fracture. (a) The protein levels of NF-*κ*B and HIF-1 in bone callus tissue were detected by western blot; (b, c) the ratio of NF-*κ*B and HIF-1 to *β*-actin protein was calculated. Compared with the NS group, ^*∗*^*P* < 0.05.

**Figure 4:** Effect of QG on BALP, BGP, and RUNX2 expressions in bone callus tissue in mice with osteoporotic fracture. (a) The protein levels of BALP, BGP, and Runx2 in bone callus tissue were detected by western blot; (b–d) the ratio of BALP, BGP, and Runx2 to *β*-actin protein was calculated. Compared with the NS group, ^*∗*^*P* < 0.05.

**Figure 5:** Effect of QG on COLI*α*1 and COLI*α*2 expressions in bone callus tissue in mice with osteoporotic fracture. (a) The protein levels of COLI*α*1 and COLI*α*2 in bone callus tissue were detected by western blot; (b, c) the ratio of COLI*α*1 and COLI*α*2 to *β*-actin protein was calculated. Compared with the NS group, ^*∗*^*P* < 0.05.

**Figure 6:** Effect of QG on the number of AVs in osteocytes in bone callus in mice with osteoporotic fracture. (a) TEM image of representative AVs in osteocytes of the three groups; (b) TEM images of osteocytes of the three groups on POD14, POD28, and POD42, with the white arrows indicating AVs; (c) AV count of the three groups on POD14, POD28, and POD42. The number of AVs was counted in each random scene under TEM scanning, and it was the mean number of AVs in osteocytes (*n* = 5) in femoral callus in each group. Compared with the NS group, ^*∗*^*P* < 0.05; compared with the ALN group, ^*#*^*P* < 0.05.

## Data Availability

The data used to support the findings of this study are available from the corresponding author upon reasonable request.
